The article "JQ1 suppresses tumor growth through downregulating LDHA in ovarian cancer" was retracted in 2026. Reasons: fabricated or falsified images; an official misconduct investigation; misconduct by an author; duplicated images.

# JQ1 suppresses tumor growth through downregulating LDHA in ovarian cancer*

**DOI:** 10.18632/oncotarget.3126

**Published:** 2015-02-05

**Authors:** Haifeng Qiu, Amanda L. Jackson, Joshua E. Kilgore, Yan Zhong, Leo Li-Ying Chan, Paola A. Gehrig, Chunxiao Zhou, Victoria L. Bae-Jump

**Affiliations:** ^1^ Department of Obsterics and Gynecology, The First Affiliated Hospital of Zhengzhou University, Zhengzhou, Henan 450052, China; ^2^ Division of Gynecological Oncology, Department of Obstetrics and Gynecology, School of Medicine, University of North Carolina at Chapel Hill, Chapel Hill, NC 27599, USA; ^3^ Division of Gynecological Oncology, Linyi Tumor Hospital, Linyi, Shandong 276001, China; ^4^ Department of Technology R&D, Nexcelom Bioscience LLC, Lawrence, MA 01843, USA; ^5^ Linberger Comprehensive Cancer Center, School of Medicine, University of North Carolina at Chapel Hill, Chapel Hill, NC 27599

**Keywords:** Ovarian cancer, BRDs inhibitor, c-Myc, Metabolism, Proliferation

## Abstract

Amplification and overexpression of c-Myc is commonly seen in human ovarian cancers, and this could be a potentially novel therapeutic target for this disease. JQ1, a selective small-molecule BET bromodomain (BRDs) inhibitor, has been found to suppress tumor progression in several cancer cell types. Using ovarian cancer cell lines, a transgenic mouse model, and primary cell cultures from human ovarian cancer tissues, we demonstrated that JQ1 significantly suppressed cellular proliferation and induced cell cycle arrest and apoptosis in ovarian cancer cells and mouse model via targeting c-Myc. In addition, JQ1 had multiple influences on cancer metabolism, particularly in the aerobic glycolysis pathway. JQ1 reduced both the activity and phosphorylation of LDHA, inhibited lactate production, and decreased the energy supply to ovarian cancer cell lines and tumors. Taken together, our findings suggest that JQ1 is an efficacious anti-tumor agent in ovarian cancer that is associated with cell cycle arrest, induction of apoptosis and alterations of metabolism.

## INTRODUCTION

Epithelial ovarian cancer is the leading cause of death from gynecological malignancies, and more than 14,000 deaths are estimated as a result of ovarian cancer in the United States this year [1]. Unfortunately, the incidence of ovarian cancer is on the rise, and more than 70% of patients will face relapse and ultimately die of their disease. The high mortality rate can be attributed to the fact that more than two thirds of patients present with late-stage disease at diagnosis, and most of them eventually develop resistance to platinum based chemotherapy. Therefore, it is urgent that we explore novel treatment approaches for ovarian cancer. Recent molecular profiling studies have shown that using small molecules to target c-Myc might be a potent strategy for ovarian cancer treatment [2, 3].

The article "JQ1 suppresses tumor growth through downregulating LDHA in ovarian cancer" was retracted in 2026. Reasons: fabricated or falsified images; an official misconduct investigation; misconduct by an author; duplicated images.

Abnormal activation of c-Myc is thought to be involved in tumor initiation and development in many types of human cancers, including breast cancer, prostate cancer, lung carcinoma, glioblastoma and ovarian cancer [4]. c-Myc is a transcription factor and functions as a DNA-binding transcriptional activator upon heterodimerization with Max to control about 30% of human genes [4, 5], which subsequently regulates the expression of multiple genes involved in cellular growth, proliferation and differentiation [6]. Knockdown of c-Myc in cancer cells *in vitro* appears to uniformly reduce cell proliferation and in some instances induce apoptosis and cell cycle arrest. In c-Myc transgenic mouse models, blocking ectopic c-Myc expression inhibits the growth of established tumors, suggesting that it is involved in tumor maintenance. Deregulation of c-Myc plays an important role in activating many transcriptional programs that influence cell division, metabolic adaptation, and survival [7, 8]. Overexpression of c-Myc often correlates with late stage cancers, poor cellular differentiation, local and distant metastases, and poor prognosis in human malignancies, including breast cancer, hepatocellular carcinoma, gastric cancer, large B-cell lymphoma, and ovarian cancer [9–14].

Previous studies using siRNA, shRNA, and small molecule inhibitors have validated the relevance of the c-Myc and its downstream genes and have proved them to be feasible therapeutic strategies for tumor treatment [8]. Several strategies have been used to target the c-Myc, including inhibition of c-Myc expression, suppression of Myc-Max dimerization, inhibition of Myc-Max DNA binding, and interference of key c-Myc related targets. JQ1 is a novel small molecule that selectively targets and inhibits actions of bromodomain-containing proteins (BRDs), thereby suppressing the tumor through the downregulation of c-Myc and its downstream targets [15]. JQ1 has been used in preclinical models with varied success in a few cancers including leukemia, glioblastoma, lung adenocarcinoma, and other malignancies [16–19].

In this study, our goal was to evaluate the potential of JQ1 on cell growth of ovarian cancer cell lines, primary ovarian cancer culture cells and an ovarian cancer mouse model. Comprehensive *in vitro* and *in vivo* studies in ovarian cancer reveal that the anti-cancer function of JQ1 affects multiple signaling pathways that regulate cell proliferation, cell cycle, apoptosis, cellular stress, metabolism, and metastasis. These results indicate that JQ1 demonstrates promise as a targeted agent for ovarian cancer.

The article "JQ1 suppresses tumor growth through downregulating LDHA in ovarian cancer" was retracted in 2026. Reasons: fabricated or falsified images; an official misconduct investigation; misconduct by an author; duplicated images.

## RESULTS

### JQ1 inhibited cell proliferation in ovarian cancer cells

We first investigated the effects of JQ1 on the growth of ovarian cancer cells and c-Myc protein expression. The ovarian cancer cell lines, Hey and SKOV3, were incubated for 72 hours with varying concentrations of JQ1. The results from the MTT assay showed a progressive decrease in cell proliferation with successive increases in the concentrations of the JQ1 (Figure 1A). After 72 hours of treatment, the IC50 of JQ1 on Hey and SKOV3 cells was 360 nM and 970 nM respectively, and the results indicated that the Hey cells were more sensitive to JQ1 than SKOV3 cells. To determine whether JQ1 effectively targets c-Myc, western blotting was performed for the Hey and SKOV3 cells after exposure to JQ1 for 24 hours. Both cell lines expressed high levels of the c-Myc protein, which was significantly suppressed by JQ1 in a dose dependent manner (Figure 1B and 1C).

**Figure 1:** JQ1 significantly suppressed growth and inhibited c-Myc expression in human ovarian cancer cell lines **(A)** JQ1 inhibited cell proliferation in a dose dependent manner after 72 hours treatment in Hey and SKOV3 cells. **(B** and **C)** The c-Myc protein was downregulated in the Hey and SKOV3 cell lines after JQ1 treatment for 24 hours (*p < 0.05; **p < 0.01).

### JQ1 induced cellular apoptosis and cell cycle arrest

In order to evaluate the cytotoxic effects induced by JQ1, ovarian cancer cells were stained with PI and Annexin V to measure the total apoptotic and necrotic cell populations. While the total apoptotic cell population (mainly the early apoptosis) increased significantly in a dose dependent manner after incubation with JQ1 for 24 hours, the necrotic cell population remained unchanged in the Hey and SKOV3 cells (Figure 2A–2C). Analysis of the different phases of the cell cycle after treatment with JQ1 demonstrated cell cycle arrest at the G1 phase. While the G1 cell population increased from 53% to 85%, the S phase decreased from 18% to 8% with increasing concentrations of JQ1 (0 to 1000 nM) in the Hey cells. Consistently, JQ1 treatment also induced G1 phase arrest and reduced S phase in the SKOV3 cell line, after 24 hours of exposure (Figure 3A–3C). To further characterize JQ1 induced cell cycle arrest, cell cycle related proteins were analyzed in JQ1 treated ovarian cancer cells. JQ1 downregulated cyclin D1, CDK4 and CDK6 protein expression and upregulated cell cycle inhibitor p21 expression in Hey and SKOV3 cells (Figure 3D and 3E). These results suggest that JQ1 inhibits ovarian cancer cell growth through the induction of apoptosis and cell cycle arrest.

The article "JQ1 suppresses tumor growth through downregulating LDHA in ovarian cancer" was retracted in 2026. Reasons: fabricated or falsified images; an official misconduct investigation; misconduct by an author; duplicated images.

**Figure 2:** JQ1 induced cellular apoptosis in a dose dependent manner JQ1 treatment induced Annexin V expression in the **(A)** Hey and **(B)** SKOV3 cell lines, within 24 hours of exposure. **(C)** Quantification of Annexin V expression (early +late apoptosis) after JQ1 treatment in the Hey and SKOV3 cell lines (*p < 0.05; **p < 0.01).

**Figure 3:** JQ1 induced cell cycle arrest in a dose dependent manner (range 0 to 1000 nM) in human ovarian cancer cell lines **(A)** JQ1 induced G1 phase arrest in the Hey cell line, after 24 hours of treatment. **(B)** JQ1 induced G1 phase arrest in the SKOV3 cell line. **(C)** Quantification of cell cycle progression after treatment with JQ1 in the Hey and SKOV3 cell lines. **(D)** After 24 hours of treatment, JQ1 increased the expression of p21 and decreased the levels of cyclin D1, CDK4 and CDK 6 in a dose dependent manner for both the Hey (the left part) and SKOV3 cell lines (the right part). **(E)** Quantification of the changes in the p21, cyclin D1, CDK4 and CDK6 proteins in the Hey and SKOV3 cell lines (*p < 0.05; **p < 0.01).

### JQ1 induced cell stress

Reactive oxygen species (ROS) have been implicated in cellular activity relating to a variety of stress responses and are involved in mediation of apoptosis via damage to the mitochondria and endoplasmic reticulum (ER). We found that JQ1 decreased the production of ROS in both cell lines in a dose dependent manner, as observed through the alterations of DCFDA fluorescence (Figure 4A). Because ROS plays a role in the induction of mitochondrial dysfunction and c-Myc regulates mitochondrial biogenesis, we also examined the effects of the JQ1 on the mitochondrial potential by JC-1 assay. We measured the mitochondrial potential (Δ ψm) by JC-1 staining in the Hey and SKOV3 cell lines after treatment with JQ1. Treatment with JQ1 for 2 hours significantly reduced the mitochondrial potential, suggesting that JQ1 specifically induces the mitochondrial dysfunction (Figure 4B). Given that treatment of tumor cells with anti-cancer agents is known to induce significant ER stress shortly after exposure. Our western blotting showed that JQ1 (500 nM) increased the expression of perk, bip and calnexin (markers for ndoplasmic reticulum stress, ER stress) as early as 3–6 hours of after treatment in the Hey and SKOV3 cells, which is further evidence of ER stress induction by JQ1 (Figure 4C–4F).

**Figure 4:** JQ1 induced cellular stress in ovarian cancer cells **(A)** JQ1 decreased the ROS level significantly in the Hey and SKOV3 cells after 24 hours treatment. **(B)** JQ1 significantly decreased the mitochondrial membrane potential in both cell lines after 2 hours treatment. **(C** to **F)** Treatment cells with JQ1 (500 nM) in time course upregulated ER stress related proteins, including perk, bip and calnexin. (*p < 0.05; **p < 0.01).

The article "JQ1 suppresses tumor growth through downregulating LDHA in ovarian cancer" was retracted in 2026. Reasons: fabricated or falsified images; an official misconduct investigation; misconduct by an author; duplicated images.

### JQ1 inhibited LDHA activity

To explore the underlying mechanism of the various cellular and molecular effects induced by JQ1 in ovarian cancer cells, we performed gene expression profiling on the Hey cell line treated with JQ1 in a time lapse manner (0, 12, 24 hours). JQ1 (500 nM) significantly impacted four specific gene groups: c-Myc and its downstream targets, apoptosis associated genes, cell cycle associated genes, and metabolism associated genes. JQ1 decreased c-Myc expression and increased p21 level as early as 12 hours after treatment, but had little influence on p27 mRNA levels. Among the cyclins and CDKs, JQ1 decreased CDK4 expression, a known downstream target of c-Myc, the most dramatically. JQ1 also increased BCL-2 and MCL-1 moderately, consistent with JQ1′s effects on induction of apoptosis (Figure 5A).

**Figure 5:** JQ1 induced transcriptomic changes in ovarian cancer cells **(A)** Four groups of genes were summarized in Hey cells based on the results of microarray analysis: c-Myc and its downstream targets (CDKN2A and CDKN2B), cell cycle associated genes (CCND1, CCND2, CDK4, CDK6 and CCNE1) and apoptosis associated genes (BCL-XL, BID, BIM, MCL1 and BCL-W). **(B)** The genes related to glycolysis and oxidative phosphorylation. JQ1 significantly affects these genes mRNA expression in Hey cells. **(C)** JQ1 decreased the expression of p-LDHA and LDHA in the Hey and SKOV3 cell lines after 24 hours treatment. **(D)** Quantification of the p-LDHA and LDHA proteins induced by the JQ1 treatment. **(E)** JQ1 inhibited LDHA activity in both ovarian cancer cell lines. **(F)** JQ1 reduced lactate production in both ovarian cancer cell lines. **(G)** JQ1 reduced ATP production in the ovarian cancer cell lines. **(H)** JQ1 reduced glucose uptake in the ovarian cancer cell lines (*p < 0.05; **p < 0.01).

In regards to the enzymes of the glycolysis pathway, LDHA (Lactate dehydrogenase A) mRNA expression decreased more substantially than the expression of other related enzymes under JQ1 treatment (Figure 5B). Given that c-Myc regulates many metabolic pathways and that JQ1 dramatically affects several genes involved in the regulation of glycolysis, we next investigated the effect of JQ1 on the functional properties of LDHA in both cell lines. The western blotting results showed JQ1 decreased the expression of LDHA and its phosphorylation after 24 hours in the Hey and SKOV3 cells, as compared to untreated cells (Figure 5C and 5D). Similarly, the enzymatic activity of LDHA and lactate production in the ovarian cancer cells was also reduced after treatment with JQ1, as evaluated by ELISA assay (Figure 5E and 5F). To further analyze the effect of JQ1 on glycolysis in ovarian cancer cells, the cellular ATP level, which is a major energy source for glycolysis in cancer cells, and glucose uptake, which is regulated by glycolysis, were assayed. We found that the ATP level and glucose uptake activity were reduced in JQ1 treated cells after 24 hours treatment (Figure 5G and 5H). These data suggest that JQ1, through inhibition of c-Myc, may be a promising glycolysis inhibitor in cancer cell metabolism.

The article "JQ1 suppresses tumor growth through downregulating LDHA in ovarian cancer" was retracted in 2026. Reasons: fabricated or falsified images; an official misconduct investigation; misconduct by an author; duplicated images.

Given that reduction of LDHA activity by siRNA and small molecule inhibitors could induce oxidative stress and cell death, we further analyzed the role of LDHA in the reduced vitality of ovarian cancer cells being treated by JQ1. We hypothesized that LDHA might be required for accentuating the inhibitive effect of JQ1, and reduced LDHA expression would increase the functional effects of JQ1 in the treatment of ovarian cancer cells. Hence, we selected a specific siRNA to block LDHA expression in Hey cells (Figure 6A). As we expected, reduction of LDHA expression with siRNA markedly decreased cell proliferation (Figure 6B). Treatment with JQ1 at 24 hours after transfection of siRNA partially increased cell viability compared with JQ1 treated cells, which is characterized by partial rescue of cell cycle processes and reduced labeling of Annexin V (Figure 6C and 6D). We then sought to determine whether reduced cellular ATP and lactate production, induced by JQ1, could be rescued by the LDHA knockdown using a specific siRNA. We found that LDHA knockdown mostly suppressed the reduction of cellular ATP and lactate levels after treatment with JQ1 for 24 hours (Figure 6E and 6F). Our results suggest that reduction of LDHA levels or activity by JQ1 triggers cell viability, and that LDHA plays an influential role in the mediation of cell proliferation and metabolism in the JQ1 treated ovarian cancer cells.

**Figure 6:** JQ1 suppressed cell growth through the downregulation of LDHA **(A)** Alterations in LDHA protein after transfection with siRNA targeting LDHA (si-LDHA) for 48 hours. **(B)** The impact of JQ1 on cell growth after treatment of si-LDHA. **(C)** The effects of JQ1 on cellular apoptosis after treatment with si-LDHA (24 hours). **(D)** The effects of JQ1 on G1 cell cycle arrest after treatment with si-LDHA (24 hours). **(E** and **F)** The effects of JQ1 on ATP and lactate production after treatment with si-LDHA (24 hours) (*p < 0.05; **p < 0.01).

### JQ1 suppressed tumor growth in orthotopic mouse ovarian cancer model

To validate the anti-tumorigenic potential of JQ1 *in vivo*, we utilized an orthotopic serous ovarian cancer mouse model by injecting M909 cells into the ovary bursa of female mice (Figure 7A). After 7–14 days of injection, palpation and autopsy confirmed ovarian cancer growth in all mice. We began JQ1 treatment (intraperitoneal injection, 50 mg/kg/day) on the mice 10–12 days after the injection of the M909 cancer cells. Tumor growth during the treatment was monitored by palpation twice a week. During the treatment, the mice showed tolerance to JQ1 injections and maintained normal activities. Regular twice-weekly measurements yielded no changes in blood glucose or weight (data not shown). After 4 weeks of treatment, the mice were euthanized, and the ovarian tumors were removed, photographed, and weighed (Figure 7B). The results showed a substantial reduction in tumor growth in the JQ1 treated group in comparison with the untreated group (Figure 7C). The JQ1 treatment group presented with tumor weights and volumes substantially lower than those of the controls (Figure 7D and 7E), indicating the efficacy of the JQ1 in ovarian cancer regression.

The article "JQ1 suppresses tumor growth through downregulating LDHA in ovarian cancer" was retracted in 2026. Reasons: fabricated or falsified images; an official misconduct investigation; misconduct by an author; duplicated images.

**Figure 7:** JQ1 significantly suppressed ovarian tumor xenograft growth and downregulated tumor glycolysis **(A** and **B)** Representative ovarian tumors from mice treated with JQ1 versus control (*n* = 8 for each group). **(C)** JQ1 significantly suppressed tumor growth. **(D)** JQ1 significantly reduced tumor weights. **(E** and **F)** JQ1 decreased the LDHA activity (* p* = 0.0015) and lactate production ( *p* = 0.028) in the ovarian tumors as compared to controls. **(G)** Immunohistochemical staining of c-Myc, LDHA, Ki 67 and cleaved caspase 3 in the ovarian tumor tissues. **(H)** Quantification of these markers in the ovarian tumor tissues (*p < 0.05; **p < 0.01; ***p < 0.001).

To further confirm the effect of JQ1 on LDHA activity *in vivo*, LDHA activity in the tumor tissues and serum lactate levels were assayed. As expected, JQ1 markedly decreased LDHA activity and lactate levels in comparison to the untreated control mice (Figure 7F). Furthermore, the expression of Ki 67, c-Myc, cleaved caspase 3 and p-LDHA were also evaluated by IHC. Consistent with our data *in vitro*, the expression of c-Myc and p-LDHA was reduced in mice treated with JQ1 but not in the untreated mice. Similarly, the levels of Ki 67 were significantly reduced following JQ1 treatment compared to the untreated controls, whereas JQ1 increased the levels of cleaved caspase 3 in treated mice (Figure 7G and 7H). As the expression of Ki 67 and cleaved caspase 3 have been correlated to cell proliferation and apoptosis, their alterations substantiated our findings that inhibition c-Myc expression by JQ1 can decrease tumor size and weight *in vivo*.

The article "JQ1 suppresses tumor growth through downregulating LDHA in ovarian cancer" was retracted in 2026. Reasons: fabricated or falsified images; an official misconduct investigation; misconduct by an author; duplicated images.

### JQ1 inhibited proliferation of ovarian cancer cells derived from patients

It is thought that primary cancer cell culture may have a stronger capability of predicting realistic drug sensitivity than immortalized cancer cell lines [20, 21]. We further investigated the effects of JQ1 on tumor cell growth in primary cultures of ovarian cancer cells by MTT assay, After 72 hours of treatment, 6 of the 7 individual patient cultures responded to the JQ1 treatment, showing an achievable IC_50_ (range from 180 nM to 1150 nM) (Figure 8A and 8B). Consistently, a decreased lactate level was detected in all six of the primary cell cultures that were sensitive to JQ1 (Figure 8C). In order to determine if the level of c-Myc protein expression was related to the sensitivity to JQ1 in ovarian cancer cells, we detected c-Myc protein expression using Western blotting in the seven untreated primary cell cultures, Hey and SKOV3 cells. The results revealed the abundant expression of c-Myc in the seven primary cultures and both the Hey and SKOV3 cells (Figure 8D, Figure 1B). An analysis of the data using a linear regression model showed that the JQ1 IC_50_ was independent upon the expression of c-Myc in the primary culture cells and both the cell lines (data not shown). These results indicate that JQ1 may be a valuable anti-cancer agent in ovarian cancer therapy.

**Figure 8:** JQ1 inhibited cellular proliferation and reduced lactate production in primary cultures of human ovarian cancer cells **(A)** The effects of JQ1 on cellular growth of the primary cultures of ovarian cancer cells, after 72 hours of exposure. **(B)** Clinical characteristics and JQ1 IC50 of these patients involved in the primary tissue culture. **(C)** Lactate production was significantly reduced in ovarian cancer cells which were sensitive to JQ1. **(D)** The expression of c-Myc protein in the seven primary ovarian cancer cells (*p < 0.05; **p < 0.01).

## DISCUSSION

Ovarian cancer is the most lethal gynecologic malignancy and ranks as the fourth most common cause of cancer-related deaths. However, there have been few improvements in ovarian cancer treatment over the last 30 years. The key to successful targeted molecular therapies against this lethal malignancy is the identification of critical, active oncogenes in oncogenic networks whose effective inhibition will result in the abrogation and/or reversal of the malignant state by induction of apoptosis and/or cellular differentiation in cancer cells. c-Myc is reported to be broadly involved in many cancers, in which its expression or amplification is estimated to be elevated or deregulated in up to 70% of human cancers [6, 22]. High levels of c-Myc expression have been linked to more aggressive ovarian cancers [13, 23]. Transgenic mouse models showed that reduced c-Myc expression resulted in tumor regression, providing evidence that tumor stability depends heavily on the activity of c-Myc. Given the fact that c-Myc is relevant to multiple cell signaling pathways that promote survival, progression, and metastasis of ovarian cancer cells, targeting c-Myc and its target genes provides a unique opportunity for ovarian cancer treatment. Recent studies have proved that activation of c-Myc could be inhibited by JQ1, a small molecule inhibitor targeting bromodomain proteins (BRDs), resulting in a remarkable inhibition of cancer cell growth and response in many cancer models in mice [24, 25].

The article "JQ1 suppresses tumor growth through downregulating LDHA in ovarian cancer" was retracted in 2026. Reasons: fabricated or falsified images; an official misconduct investigation; misconduct by an author; duplicated images.

Inhibition of c-Myc by small molecular inhibitors has been investigated in cancer therapeutics over last several years, but to date, due to low potency or efficiency, no inhibitors have been effectively incorporated into routine chemotherapies. The present study is the first to demonstrate that JQ1 reduces the viability of ovarian cancer cells and primary cultured ovarian cancer cells by inducing apoptosis (through the downregulation of MCL-1 and BCL-2), cell cycle arrest (through upregulation of p21 and p27, downregulation of cyclin D1, CDK4 and CDK6), and by inhibiting ovarian cell migration and metabolism. By decreasing c-Myc expression in our orthotopically transplanted serous ovarian cancer mouse model, JQ1 ultimately led to a decrease in tumor volume, following reduction in Ki 67 expression and an increase in cleaved caspase 3 levels.

One of the hallmarks of cancer cells is an increased dependence on glycolytic metabolism and the production of large quantities of lactate regardless of oxygen availability, which is known as the Warburg effect [26, 27]. It is featured by the high flux of glucose into tumor cells even in a non-hypoxic microenvironment, ending with the conversion of pyruvate into lactate and resulting in a high production of lactate to generate sufficient energy for the demands of rapidly proliferating tumor cells [28–30]. Based on previous reports, c-Myc appears to be an important transcription factor for glucose metabolism both in normal and cancer tissues [7, 31]. Overexpression of c-Myc induces the expression of glycolytic enzymes such as lactate dehydrogenase-A (LDHA), glucose transporter-1 (GLUT1), hexokinase-2 (HK2) and increases glycolysis in most cancer cells [32]. In our study, JQ1 significantly decreased cellular glucose uptake and ATP and lactate production in ovarian cancer cells. Metabolic alterations may also play a crucial role in chemoresistance in patients with ovarian cancer [33], and future studies will be focused on whether JQ1 may aid in overcoming chemoresistance in this disease. In addition, the targeting of key control points of glycolysis is emerging as a novel strategy in regards to cancer therapy, further supporting the use of JQ1 which is able to target both proliferative and metabolic pathways.

The article "JQ1 suppresses tumor growth through downregulating LDHA in ovarian cancer" was retracted in 2026. Reasons: fabricated or falsified images; an official misconduct investigation; misconduct by an author; duplicated images.

Among the glycolytic enzymes, lactate dehydrogenase A (LDHA) is unique as it is essential to maintain the rapid regeneration of NAD+ [34]. The upregulated expression and activity of LDHA has been detected in breast cancer, pancreatic cancer, melanoma and ovarian cancer and has been significantly associated with poor prognosis [35–39]. In both *in vitro* and *in vivo* studies, silencing LDHA by either RNA interference or small molecule inhibitors has been found to significantly suppress tumor initiation and progression [40, 41]. Given that most normal tissues are not LDHA(lactate)-dependent, targeting LDHA is proposed to be a promising therapeutic strategy for specifically targeting cancer cells over normal cells [41, 42]. Previously, c-Myc had been found to be able to activate the transcription of LDHA via binding to the Myc/Max binding sites located in the promoter of LDHA [43]. In regards to our microarray data, JQ1 significantly inhibited LDHA mRNA expression, which subsequently reduced phosphorylation of LDHA and LDHA activity. Knockdown of LDHA was shown to eliminate the suppressive effects of JQ1 on cancer cell proliferation and glycolysis. More importantly, JQ1 treatment not only reduced tumor growth but also decreased LDHA activity and lactate levels in our mouse model. The correlation between JQ1 treatment and LDHA activity has been documented recently by other research groups via genome-wide expression profiling analysis in acute lymphoblastic leukemia [44]. Taken together with other studies, our results support that beyond its anti-proliferative properties, JQ1 is an effective inhibitor of glycolysis through the targeting of LDHA, a key rate limiting enzyme of glycolysis in ovarian cancer [32, 45].

It is thought that primary cancer cell culture, in evaluating the efficacy of anti-cancer agents, has greater sensitivity than cancer cell lines and provides high-fidelity data for translating *in vitro* findings into clinical settings [20, 21]. In a panel of 7 primary cell cultures from serous ovarian cancer patients, 6 cases showed diverse ranges of IC50 (180–1150 nM) and relatively decreased lactate levels after 72 hours of JQ1 treatment, providing further support for the use of JQ1 as a targeted therapy for ovarian cancer.

The article "JQ1 suppresses tumor growth through downregulating LDHA in ovarian cancer" was retracted in 2026. Reasons: fabricated or falsified images; an official misconduct investigation; misconduct by an author; duplicated images.

Potent cytotoxicity and efficacy of JQ1 toward a wide range of cancer cell lines and *in vivo* pre-clinical models has been extensively investigated worldwide, making JQ1 an attractive candidate for further investigation as a potential anti-cancer agent in clinical trials in the near future, including that of ovarian cancer based on our studies. A deeper understanding of the underlying molecular mechanisms of JQ1′s anti-tumorigenic activity will allow for more tailored treatment regimens and the possibility to combine JQ1 with other complementary cytotoxic and targeted therapeutics to achieve the most synergistic results in tumor regression.

## MATERIALS AND METHODS

### Ovarian cancer cell lines and reagents

The medium were RPMI 1640 with 5% fetal bovine serum for Hey and M909, and DMEM/F12 with 10% fetal bovine serum for SKOV3. Hey and SKOV3 were purchased from ATCC (American type culture collection, USA). The M909 cell line was established in our laboratory from the T_121+_ p53^f/f^ Brcar1^f/f^ serous ovarian cancer mouse model [46]. These cell lines were cultured under standard conditions at 37°C in a humidified incubator containing 5% CO_2_. JQ1 was a kindly gift by Dr. James E. Bradner (Harvard medical school, MA, USA). The non-fat milk, 20% bull serum albumin (BSA) and RNase A were purchased from Sigma (St. Louis, MO, USA ), and all the primary antibodies for c-Myc, LDHA, p-LDHA, cyclin D1, CDK4, CDK6, p21, p27, Ki 67, cleaved caspase 3, perk, bip, calnexin and α-tubulin were obtained from Cell Signaling Technology (Danvers, MA, USA).

### Ovarian cancer tissue samples collection and primary cell culture

Seven tumor specimens were sampled from patients undergoing surgery for serous ovarian carcinoma at the University of North Carolina at Chapel Hill (UNC-CH). The protocol was reviewed and exemption granted by the Institutional Review Board at UNC-CH. Tumors were staged and graded according to the criteria of the International Federation of Obstetrics and Gynecology (FIGO, 2009). For the culture of primary ovarian cancer cells, the freshly obtained tissues were washed three times with Hank's Buffered Salt Solution (HBSS), and then gently minced by scissors in DMEM/F12 medium containing 10% fetal bovine serum (FBS). These tissues were then digested in 0.2% collagenase IA, 100 U/ml penicillin and streptomycin for 30–60 minutes at 37°C water bath with shaking. After two centrifugations with PBS solution, cells were re-suspended and diluted to 1 × 10^5^ cells/ml with DMEM/F12 medium. Subsequently, 1 × 10^4^ cells/well were seeded into 96-well plates and incubated for 24 hours before JQ1 treated. Cell proliferation was measured by MTT assay 72 hours after JQ1 treatment.

The article "JQ1 suppresses tumor growth through downregulating LDHA in ovarian cancer" was retracted in 2026. Reasons: fabricated or falsified images; an official misconduct investigation; misconduct by an author; duplicated images.

### Proliferation assay

The impact of JQ1 on the cellular proliferation of Hey, SKOV3 and primary culture of human ovarian cancer cells was determined by MTT assay. Briefly, 4 × 10^3^ cells/well were seeded into 96-well plates and incubated overnight with the indicated medium, then treated with different doses of JQ1 (from 0 to 10000 nM) for 72 hours. Subsequently, 5 μl MTT (5 mg/ml; Sigma, St. Louis, MO, USA) was added into each well and incubated for 1 hour. The MTT reaction was terminated by the addition of 100 μl DMSO. The results were determined by measuring the absorbance at 570 nm with a microplate reader (Tecan, Morrisville, NC, USA). The effect of JQ1 was calculated as a relative percentage of control cell growth obtained from DMSO (0.1%) treated cells grown in the same 96-well plates. Each experiment was performed in triplicate and repeated three times to assess for consistency of results.

### Western blot analysis

Total protein was extracted from ovarian cancer cells or tissues using RIPA buffer (Thermo Fisher, MA, USA) and quantified with the BCA assay kit (Thermo Fisher). Equal amounts (30–50 μg) of total protein were loaded and separated by 10–12% SDS-PAGE, then transferred to PVDF membrane, blocked in 5% non-fat milk and incubated with the primary antibodies overnight at 4°C. Subsequently, the membranes were incubated with the appropriate secondary antibodies for 1 hour at room temperature before development. The bands were developed and quantified using an Alpha Innotech Imaging System (San Leandro, CA, USA). After developing, the membranes were stripped or washed and re-probed using antibodies against total LDHA (for p-LDHA) and α-tubulin (for all proteins), respectively. Each experiment was repeated three times to assess for consistency of results. α-tubulin was used as the endogenous control.

### Cell cycle analysis

The effect of JQ1 on the cell cycle was measured using Cellometer (Nexcelom, Lawrence, MA, USA). Briefly, 2.5 × 10^5^ cells/well were seeded into 6-well plates and incubated overnight, then treated with JQ1 (from 0 to 1000 nM) for 24 hours. The cells were harvested and washed with phosphate buffered saline (PBS), the pellet was re-suspended and fixed in 90% pre-chilled methanol and stocked overnight at −20°C. The cells were then washed with PBS again and re-suspended in 50 μl RNase A solution (250 μg/ml, 10 mM EDTA) for 30 minutes and then 50 μl staining solution [containing 2 mg/ml PI (Biotium, Hayward, MA, USA), 0.1 mg/ml Azide (Sigma), and 0.05% Triton X-100 (Sigma)] was added into. The final mixture was incubated for 15 minutes in dark before analyzed on Cellometer. The results were analyzed using FCS4 express software. The experiments were performed in triplicate and repeated three times.

The article "JQ1 suppresses tumor growth through downregulating LDHA in ovarian cancer" was retracted in 2026. Reasons: fabricated or falsified images; an official misconduct investigation; misconduct by an author; duplicated images.

### Apoptosis assay

JQ1 induced apoptosis was detected with PI/Annexin V staining kit (Biolegend, San Diego, CA, USA). Briefly, 2.5 × 10^5^ cells/well were seeded into 6-well plates and incubated overnight, then treated with JQ1 (from 0 to 1000 nM) for 24 hours. The cells were then collected, washed with PBS, and re-suspended in the 100 μl binding buffer. One μl of Annexin V and 0.5 μl of propidium iodide (10 mg/ml) were added in the binding buffer for 15 minutes in the dark. The samples were immediately measured by Cellometer. The results were analyzed by FCS4 express software. The total apoptotic cells (early apoptosis+late apoptosis) were expressed as a percentage of the total number of cells stained. All experiments were performed in triplicate and repeated three times to assess for consistency of response.

### Mitochondrial membrane potential measurement

JC-1 (5,5′,6,6′-tetrachloro-1,1′,3,3′-tetraethylbenzimidazolcarbocyanine iodide, Invitrogen, Grand Island, NY, USA) was used to detect changes of the mitochondrial membrane potential. 1 × 10^6^ cells/well were seeded into 6-well plates and incubated overnight, then the cells were treated with JQ1 for 2 hours and stained with JC-1 (200 μM) for 15 minutes in the dark, and measured by Cellometer. The results were analyzed by FCS4 express software. All experiments were performed in triplicate and repeated three times.

### RNA interference experiments

siRNAs targeting human LDHA (SI00078897) were purchased from Qiagen Company (Hilden, Germany). Transfection of siRNAs was performed using the Qiagen Hiperfect transfection reagent according to the manufacturer's instructions. Briefly, 1 × 10^6^ cells/well were seeded into the 6-well plates and incubated overnight, and then a mixture consisting of 75 ng of si-LDHA and 5 μl Qiagen Hiperfect was added into the medium. 48 hours later, the cells were harvested for western blot and other assays. A scramble siRNA was used as the negative control. The experiments were repeated in triplicate.

### Lactate production assay

Lactate production in the medium was detected by using the Lactate Assay Kit (BioVision, Mountain View, CA, USA). Briefly, at the finish of JQ1 treatment, 2 μl corresponding medium was taken for the lactate assay. The medium was mixed with reaction buffer and incubated for 30 minutes at 37°C in the dark. Fluorescence was then measured at Ex/Em = 535/587 nm on a microplate reader. Results were normalized on the basis of the total protein concentration of each sample. All the experiments were performed in triplicate and repeated twice.

The article "JQ1 suppresses tumor growth through downregulating LDHA in ovarian cancer" was retracted in 2026. Reasons: fabricated or falsified images; an official misconduct investigation; misconduct by an author; duplicated images.

### LDHA activity assay

Alterations of cellular LDHA activity were determined using the LDHA Activity Assay Kit (BioVision), following the manufacturer's instructions. Briefly, 2 × 10^5^ cells/well were seeded into 6-well plates and incubated overnight, then treated with JQ1 (from 0 to 1000 nM) for 24 hours. Cells were lysed with the cold assay buffer and centrifuged at 10,000 × g for 15 minutes at 4°C. 5 μl supernatant was then mixed with 45 μl reaction buffer. The absorbance (450 nm) was measured at 0 minutes (T_1_) after 30 minutes of incubation at 37°C (T_2_), using a plate reader. The relative LDHA activity was determined by (T_2_–T_1_). All results were normalized on the basis of the total protein concentration of the cells. All the experiments were performed in triplicate and repeated three times.

### Measurement of ATP

ATP production was determined using the luminometric ATP assay kit (AAT bioquest, Sunnyvale, CA, USA) following the manufacturer's instructions. In brief, 5 × 10^3^ cells were seeded in 96-well plates and incubated overnight, followed by the treatment with different doses of JQ1 for 24 hours. Then, 100 μl/well ATP assay solution was added into and mixed gently, incubate for 20 minutes at room temperature. The luminescence intensity was measured in luminometer mode on a plate reader. Finally, all the results were normalized on the basis of the total protein derived from the cells treated exactly as the ATP group. The experiments were performed in triplicate and repeated three times.

### Glucose uptake assay

The glucose uptake assay was performed using 2-[N-(7-nitrobenz-2-oxa-1,3-diazol-4-yl)amino]-2-deoxy-D-glucose (2-NBDG; Invitrogen), followed by detection of fluorescence produced by the cells [45]. 24 hours after treated with JQ1, the Hey and SKOV3 cells were incubated with 2-NBDG (100 μM) with glucose free medium for 15 minutes. The 2-NBDG uptake reaction was stopped by removing the medium and washing the cells twice with 200 μl HBSS. Fluorescence (excitation/emission [Ex/Em] = 485/535) was measured using the plate reader. Relative glucose was assayed compared with untreated control. All the experiments were performed in triplicate and repeated three times.

### Reactive oxygen species (ROS) assay

The Fluorimetric Intracellular Total ROS Activity Assay Kit (AAT bioquest) was used to detect the alteration of total production of reactive oxygen species caused by JQ1. Briefly, 1 × 10^4^ Hey and SKOV3 cells were pre-stained by the ROS working solution for 1 hour and then treated by JQ1 for 30 minutes. The fluorescence was monitored at Ex/Em = 490/525 nm on the plate reader. All the experiments were performed in triplicate and repeated three times.

The article "JQ1 suppresses tumor growth through downregulating LDHA in ovarian cancer" was retracted in 2026. Reasons: fabricated or falsified images; an official misconduct investigation; misconduct by an author; duplicated images.

### Orthotropic xenografts of serous ovarian cancer

The vast majority of epithelial ovarian tumors are of the serous histologic type (75–80%). The K18-gT_121_^+/–^; p53^fl/fl^; –Brca1^fl/fl^ (KpB) mouse model is a unique serous ovarian cancer mouse model that specifically and somatically deletes the tumor suppressor genes, Brca1 and p53, and inactivates the retinoblastoma (Rb) proteins in adult ovarian surface epithelial cells (KpB mouse model) [8]. At 4–6 months, tumors develop in the affected ovary, while the un-injected ovary remains normal and can be used as a contralateral control. Histologic examination and marker studies demonstrate that the KpB ovarian tumors recapitulate the major features of serous ovarian cancer. As an extension of this model, we have established an ovarian tumor cell line from one of the KpB mice (M909). Upon re-injection of these tumor cells into the ovarian bursa of female mice, we have developed a more aggressive variant of the KpB model. At 10–14 days after injection of these tumor cells, a tumor can be palpated on the ovary of these mice. At 28–42 days, all of these mice have disseminated disease throughout the abdomen (unpublished data).

For the evaluation of JQ1′s *in vivo* effects, M909 cells (1 × 10^6^ cells/5 μl) were injected into left side of the ovarian bursa of 6–8 week old T_121+_ p53^f/f^ Brcar1^f/f^ female mice. All mice were handled according to protocols approved by UNC-CH Institutional Animal Care and Use Committee (IACUC). Twenty mice were injected with the M909 cells and then randomly divided into the control, placebo (saline) group and JQ1 treatment group. The JQ1 treatment (intraperitoneal injection, 50 mg/kg/day) was initiated twelve days after the injection, and the tumor was palpated twice a week, when tumor reached certain size (more than 0.4–0.5 cm), we measured the tumor by calipers twice a week. Tumor volume was calculated using the following equation: tumor volume = (width2 × length)/2. All mice were euthanized after four weeks of JQ1 or placebo treatment. Tumor tissue and blood samples were collected for immunohistochemical staining, measurement of LDHA activity and lactate production assays.

### Microarray analysis

2.5 × 10^5^ Hey cells/well were seeded into 6-well plates and incubated overnight and then treated with JQ1 for 0, 6, 12, 24 hours. Total RNA was extracted from cells using the RNAeasy Kit (Qiagen). RNA integrity was measured on the Agilent 2100 Bioanalyzer. Total RNA amplification and labeling were done as previously described [47]. The hybridization was performed using Agilent 244K Human oligonucleotide microarrays. The results were analyzed with GenePix Pro 4.1 and uploaded onto the Microarray Database of UNC-CH.

The article "JQ1 suppresses tumor growth through downregulating LDHA in ovarian cancer" was retracted in 2026. Reasons: fabricated or falsified images; an official misconduct investigation; misconduct by an author; duplicated images.

### Immunohistochemical analysis

The mouse tumor tissue was formalin-fixed and paraffin-embedded. Slides (5 μm) were first incubated with Protein Block solution (Dako) for 1 hour and then with the primary antibodies for c-Myc (1: 200), LDHA(1: 200), Ki-67(1: 400) and cleaved caspase-3(1: 300) for 2 hours at room temperature. The slides were then washed and incubated with appropriate secondary antibodies at room temperature for 1 hour. The slides were washed, and the specific staining was visualized using the SignalStain Boost IHC Detection Reagent (Cell Signaling Technology) following the manufacturer's instructions. Individual slides were scanned using the Aperio™ ScanScope (Aperio Technologies, Vista, CA), and digital images were analyzed for target protein expression using Aperio™ ImageScope software.

### Statistical analysis

Results were compared by Student's *t* test and data were expressed as mean ± S.E. Statistical significance was defined to be *p* < 0.05.
